This article has been retracted.

# Predictive Significance of High-Sensitivity C-Reactive Protein Combined with Homocysteine for Coronary Heart Disease in Patients with Anxiety Disorders

**DOI:** 10.1155/2022/7657347

**Published:** 2022-08-23

**Authors:** Changhe Liu, Na Hua, Yanli Zhang, Cuirong Wang

**Affiliations:** ^1^Department of Cardiology, Affiliated Zhongshan Hospital of Dalian University, Dalian 116001, China; ^2^Department of Otolaryngology, Affiliated Zhongshan Hospital of Dalian University, Dalian 116001, China; ^3^Department of Neurology, Affiliated Zhongshan Hospital of Dalian University, Dalian 116001, China

## Abstract

**Background:**

Currently, there are few studies on biomarkers for predicting coronary heart disease (CHD) with anxiety disorders.

**Objective:**

To explore risk factors and investigate the predictive value of common clinical peripheral blood indicators, such as high-sensitivity C-reactive protein (hs-CRP) and homocysteine (Hcy) for CHD patients with anxiety disorders.

**Methods:**

One hundred fifty-three hospitalized patients with chest pain as the main symptom and a Hamilton Anxiety Scale score > 14 were recruited from October 2020 to September 2021 in the hospital. Then, they were divided into an anxiety disorder with CHD group (observation group, *n* = 64) and a simple anxiety disorder group (control group, *n* = 89), according to coronary angiography (CAG) findings. Patients' demographic and clinical messages were collected and compared. Diabetes mellitus and hypertension, body mass index (BMI), and peripheral blood interleukin-6 (IL-6), high-sensitivity C-reactive protein (hs-CRP), homocysteine (Hcy), fibrinogen, D-dimer, cortisol, and norepinephrine expression levels were compared. Binary logistic regression analysis screened independent risk factors of CHD patients with anxiety disorders. The effectiveness of independent risk factors in predicting CHD with anxiety disorders was analyzed using receiver operating characteristic (ROC) curves.

**Results:**

IL-6, hs-CRP, and Hcy levels of anxiety disorder in the CHD group were significantly higher than those in the simple anxiety disorder group. Binary multiple logistic regression analysis indicated that IL-6, hs-CRP, and Hcy were independent risk factors for CHD in patients with anxiety disorders. hs-CRP and Hcy levels were positively correlated with the Gensini score. ROC curve analysis indicated that the detection of hs-CRP or Hcy alone or the combined detection of the 2 had clinical predictive value for CHD in patients with anxiety disorders, and the area under the curve (AUC) of the combined detection of the 2 was significantly larger than that of any single factor alone (vs. hs-CRP, *P* = 0.045; vs. Hcy, *P* = 0.045).

**Conclusion:**

IL-6, hs-CRP, and Hcy are related to CHD with anxiety disorders. Serum levels of the combined detection of hs-CRP and Hcy have a high clinical predictive value for CHD in patients with anxiety disorders.

## 1. Background

According to WHO statistics, coronary heart disease is the most common cause of death in the world, and 81% of the main causes of sudden cardiac death are coronary heart disease (CHD) [1, 2]. Among the patients with cardiovascular disease in China, CHD ranks second only to stroke. In recent years, with the improvement of living standards and lifestyle changes, the incidence of coronary heart disease has significantly increased, which seriously affects people's health and life safety [3]. CHD is a narrowing of the vascular cavity caused by atherosclerotic coronary arteries, which can cause heart disease due to myocardial necrosis, hypoxia, and ischemia. Currently, the main pathogenic factors of CHD include abnormal blood sugar, hyperlipidemia, smoking, obesity, hypertension, and altitude [4]. At this stage, the main method of clinical treatment of CHD is to improve the blood supply speed of the coronary artery in the patient, so that the myocardial oxygen consumption of the patient can be reduced, thereby improving the clinical symptoms of the patient. CHD has become an important disease affecting people's physical and mental health. Studies have shown that CHD is connected with anxiety disorders [5, 6]. Psychocardiological abnormality has gradually become an important pathogenesis of CHD and a popular topic in cardiovascular disease research.

CHD is a typical psychosomatic disease. Patients are prone to negative emotions such as anxiety during the disease course. A previous study showed that people with anxiety disorders in the CHD population are 11%, significantly higher than the incidence (3%-7%) of anxiety disorders in the general population [7]. Moreover, the incidence of CHD with anxiety is increasing worldwide, and CHD with anxiety is characterized by high mortality and poor prognosis [8]. In addition, long-term anxiety can promote or aggravate CHD, adversely affecting the treatment compliance, drug efficacy, and prognosis of patients [9]. Anxiety disorder has been confirmed as a CHD risk factor, thus increasing CHD risk in the general population [5] and serving as an important basis for the prognostic assessment of CHD [10].

The physical symptoms of CHD and anxiety disorder (such as chest pain, dizziness, dyspnea, palpitations, and fatigue) significantly overlap [11, 12]. Clinically, patients with chest pain as the main manifestation and treated in cardiovascular medicine departments not only have a high rate of missed anxiety disorder diagnosis but are also easily confused with angina pectoris. Due to the characteristics of anxiety, some patients strongly refuse coronary angiography (CAG), which causes difficulties in diagnosing and treating CHD. On the other hand, some patients with anxiety disorders strongly demand CAG, which increases the incidence of complications and constitutes a waste of medical resources. Therefore, it is vital to strengthen the identification of noninvasive biomarkers in patients with anxiety disorders complicated by CHD.

Currently, biomarkers for predicting CHD in the general population are of more clinical concern, but there are few studies on biomarkers for predicting CHD in the population with anxiety disorders. The aim is to investigate the predictive value of common clinical peripheral blood indicators, such as interleukin-6 (IL-6), high-sensitivity C-reactive protein (hs-CRP), and homocysteine (Hcy), in patients with anxiety disorders and to explore CHD risk factors of anxiety disorder patients. Understanding these helps to identify a high-risk CHD patient among anxiety disorder patients and guide clinical treatment strategies.

## 2. Patients and Methods

### 2.1. Patients

The Ethics Committee approved the study protocol of the Affiliated Zhongshan Hospital of Dalian University (No. 2021046). Written informed consent to participate in the study was given to all patients.

This cross-sectional study was a single-center, prospective study at the Department of Cardiology from October 2020 to September 2021 (Registration Number: ChiCTR2200057008). This study applied the Hamilton Anxiety Scale (HAMA) to evaluate anxiety in hospitalized cardiology patients with chest pain. Patients with anxiety disorders (HAMA score > 14) were included as research participants. CAG was performed if needed, and coronary artery stenosis greater than 50% was identified as CHD. Then, the study participants were divided into an anxiety disorder with CHD group and a simple anxiety disorder group. All patients completed the study, and no patient dropped out of the study.

### 2.2. Inclusion and Exclusion Criteria

Inclusion criteria are as follows: (1) age > 18 years old and an education level of elementary school or above and (2) HAMA score > 14 and CAG completed during hospitalization.

Exclusion criteria are as follows: (1) a clear history of mental illness; (2) acute myocardial infarction; (3) a clear diagnosis or denial of CHD; (4) a history of arrhythmia, heart failure, autoimmune disease, stroke, liver or kidney dysfunction, thyroid dysfunction, structural heart disease, or malignant tumors; (5) a history of infectious diseases within the past 3 months; (6) a history of taking hormones, folic acid, or vitamin B12 within the past 3 months; and (7) patients without complete clinical data.

### 2.3. HAMA Assessment

HAMA is used for anxiety disorder diagnosis and determining its severity [13]. It has high reliability and validity. The scale has 14 items that address anxiety, tension, insomnia, paresthesia, depression, physical anxiety, etc., with each item scored using a 5-level (0-4) scoring method. A higher total score means severe anxiety. Scores less than 7, 7-14, greater than 14 and no greater than 21, greater than 21 and no greater than 29, and greater than 29 indicate no anxiety, possible anxiety, definite anxiety, considerable anxiety, and severe anxiety, respectively. The psychologists in our hospital evaluated patients with this scale at the time of admission and recorded their HAMA scores. Patients' HAMA scores should be >14.

### 2.4. Risk Factors

Gender, age, smoking status, diabetes mellitus, hypertension, body mass index (BMI), and peripheral blood IL-6, hs-CRP, Hcy, fibrinogen, D-dimer, cortisol, norepinephrine, total cholesterol, high-density lipoprotein cholesterol (HDL-C), low-density lipoprotein cholesterol (LDL-C), triglyceride, lipoprotein (a), apolipoprotein B, and creatinine expression levels were used to analyze CHD risk factors in anxiety disorder patients.

### 2.5. Laboratory Examinations

They have collected fasting venous blood. Within 1 hour after collection, the blood sample was centrifuged (3000 rpm, 15 minutes), and the serum was stored at 2-8°C. Serum IL-6 levels were measured by chemiluminescence microparticle immunoassay (Caris 200; Wantai Biopharm, Beijing, China). Serum hs-CRP and Hcy levels were detected by latex immunoturbidimetry (Abbott ARCHITECT® System, Architect -c16000; Abbott, TX, USA). Serum levels were determined (Abbott ARCHITECT® System, Architect-i 2000; Abbott, TX, USA) by chemiluminescence microparticle immunoassay. Additionally, an automatic biochemical analyzer was used to measure the levels of blood fibrinogen, D-dimer, cortisol, HDL-C, LDL-C, creatinine, and other biochemical indicators.

### 2.6. Gensini Score

The Gensini score is an evaluation standard for assessing coronary artery stenosis degree, accurately reflecting CHD severity. Based on the CAG report, the degree of stenosis in each coronary artery was quantitatively assessed. The degree of vascular stenosis was scored as follows: 100%, 32 points; 91%-99%, 16 points; 76%-90%, 8 points; 51%-75%, 4 points; 26%-50%, 2 points; and ≤25%, 1 point. The scores were multiplied by the corresponding coefficients for the coronary branches. The coefficients were 5 for the left main artery; 2.5 for the proximal segment of the anterior descending branch and the proximal segment of the circumflex branch; 1.5 for the middle segment of the anterior descending branch; 1 for the distal segment of the anterior descending branch, the right coronary artery, the distal segment of the circumflex branch, the first diagonal branch, the first obtuse marginal branch, and the posterior descending branch; and 0.5 for the remaining branches. The Gensini score is the sum of each vascular stenosis score multiplied by the corresponding coefficient. A higher Gensini score denotes severe coronary stenosis.

### 2.7. Statistical Analysis

SPSS 26.0 was used for statistical analysis. Categorical variables were specified as *n* (%). A chi-square test compared proportions in the different groups. Independent sample *T*-test or Mann–Whitney *U* test compared the groups. The Spearman correlation test analyzed the correlation coefficient and its significance. Binary logistic regression analysis determined CHD risk factors in patients with anxiety disorders. The area under the receiver operating characteristic (ROC) curve (AUC) was calculated to investigate the predictive significance of relevant risk factors for CHD in patients with anxiety disorders. The *Z* test was performed using MedCalc19 software to compare the differences in AUC. *P* < 0.05 was considered statistically significant.

## 3. Results

### 3.1. Patient Information

One hundred fifty-three participants were in this research. Among them, there were 64 patients in the anxiety disorder with CHD group (observation group) and 89 patients in the simple anxiety disorder group (control group). Clinical data and laboratory indicators are shown in Table 1. There has been no change in HAMA score, BMI, or the expression levels of fibrinogen, D-dimer, cortisol, norepinephrine, total cholesterol, HDL-C, LDL-C, triglyceride, lipoprotein (a), apolipoprotein B, and creatinine between the anxiety disorder with CHD and simple anxiety disorder groups. The proportion of male patients, age, the smoked proportion, the diabetes proportion, the hypertension proportion, the elevated IL-6, and the serum hs-CRP and Hcy level proportion of CHD with anxiety disorder group was significantly higher than that of the simple anxiety disorder group (*P* <0.05) (Table 1).

### 3.2. Risk Factors of CHD Combined with Anxiety Disorders

Univariate logistic regression analysis determines the risk factors of CHD combined with anxiety disorders. The following were significantly different between the anxiety disorder with CHD group and the simple anxiety disorder group: sex (*P* = 0.004), age (*P* = 0.031), smoking status (*P* = 0.005), diabetes mellitus (*P* = 0.008), hypertension (*P* = 0.005), and IL-6 levels (*P* < 0.001), hs-CRP (*P* < 0.001), and Hcy (*P* < 0.001); the other variables have no change (Table 2).

### 3.3. Binary Multiple Logistic Regression Analysis of Risk Factors for CHD with Anxiety Disorders

We included risk factors in univariate analysis, namely, sex, age, smoking status, diabetes mellitus, hypertension, and hs-CRP, Hcy, and IL-6 levels in our binary multiple logistic regression model to evaluate their predictive significance for CHD in patients with anxiety disorders. Analysis indicated that hs-CRP (odds ratio (OR) 1.386, 95% CI 1.156–1.662, *P* = 0.017), Hcy (OR 1.220, 95% CI 1.101–1.351, *P* = 0.006), and IL-6 (≥3.5 pg/mL vs. <3.5 pg/mL: OR 0.154, 95% CI 0.064–0.373, *P* = 0.001) were independent risk factors for CHD in patients with anxiety disorders after adjusting sex, age, smoking status, diabetes mellitus, and hypertension (Table 2).

### 3.4. Spearman Correlation Analysis

Analysis was performed for serum hs-CRP levels and Gensini scores and for Hcy levels and Gensini scores. The results showed that serum hs-CRP and Hcy levels were positively correlated with the Gensini score (*r* = 0.278, *P* = 0.001; *r* = 0.374, *P* < 0.001), indicating that both indicators were reliable.

### 3.5. ROC Analysis

ROC curves were constructed to obtain the optimal cutoff value and predict the risk for coronary heart disease in anxiety disorder patients (Figure 1). AUC is used to measure the reliability of the model, in which a value close to 1.0 indicates high diagnostic accuracy. The results showed that the optimal cutoff values with the greatest sensitivity and specificity for predicting CHD in patients with anxiety disorders were 2.00 mg/L (sensitivity, 0.47; specificity, 0.88) for hs-CRP and 11.96 *μ*mol/L (sensitivity, 0.48; specificity, 0.85) for Hcy. The AUC was 0.669 (95% CI 0.580-0.758, *P* < 0.001) for hs-CRP and 0.684 (95% CI 0.597-0.771, *P* < 0.001) for Hcy. The AUC for combined detection of hs-CRP and Hcy was 0.749 (95% CI 0.671-0.827, *P* < 0.001). Interestingly, we found that the combined detection of the 2 can better predict whether patients with anxiety disorders have CHD than the detection of hs-CRP or Hcy alone [vs. hs-CRP (*Z* = 2.006, *P* = 0.045); vs. Hcy (*Z* = 2.003, *P* = 0.045)] (Figure 1).

## 4. Discussion

We focused on the predictive significance and effectiveness of peripheral blood biomarkers in patients with anxiety disorders. We found that IL-6, hs-CRP, and Hcy serum levels were CHD-independent risk factors for anxiety disorder patients, which still had predictive value. Patients with anxiety disorders complicated with CHD had higher IL-6, hs-CRP, and Hcy levels than did simple anxiety disorder patients. Our data provide a noninvasive clinical prediction of CHD in anxiety disorder patients and have positive clinical guidance value.

Inflammatory biomarkers are indicators of the pathogenic process or pharmacological response [14]. CHD is an important cause of high mortality worldwide. One of the most common causes of CHD is atherosclerosis-related vascular inflammation [15], and the inhibition of inflammation can significantly reduce the recurrence rate of atherosclerotic diseases [16]. Currently, inflammatory biomarkers can be used to aid in the detection of cardiovascular diseases and to monitor their evaluation, prognosis, and treatment progress [17, 18]. Although increasing evidence has shown that CHD and anxiety disorders are associated with inflammatory biomarkers, few studies have focused on the predictive peripheral blood inflammatory biomarkers for CHD in anxiety disorder patients. This study focuses on the predictive value of peripheral blood biomarkers for CHD in patients with anxiety disorders.

IL-6 is a multipotent immunomodulatory cytokine secreted by activated macrophages, lymphocytes, and fat cells that play an essential role in many inflammatory processes [19]. IL-6 expression is associated with atherosclerosis, and IL-6 is an inflammatory cytokine closely related to CHD [20]. Clinical studies have found that IL-6 expression is significantly elevated in the serum of patients with CHD [18] and increases the incidence of myocardial infarction and cardiovascular death as well as the rate of cardiac hospitalization and all-cause mortality [21]. As an acute-phase protein produced by proinflammatory cytokines, CRP, which promotes the uptake of oxidized LDL-C by macrophages and accelerates the process of atherosclerosis, is another important inflammatory biomarker. CRP is an important cardiovascular disease risk factor [22] and can be used as a biomarker for cardiovascular disease prognosis [22]. Studies have confirmed that elevated hs-CRP is connected with coronary endothelial dysfunction, plaque formation, and coronary stenosis and is an abnormal coronary vascular response independent predictor [23, 24]. Inflammatory cells stimulated by inflammatory cytokines can promote the production of IL-6, leading to the massive synthesis of hs-CRP in the liver [25]. There is correlation between the circulating concentrations of IL-6 and CRP. IL-6 may act upstream of CRP to regulate CRP expression [26, 27], and CRP can reflect the status of IL-6 secretion [28]. In summary, as an essential systemic inflammatory mediator, IL-6 can promote the elevation of CRP levels and further increase the risk of CHD [26].

Anxiety disorders are the most common mental disorders with a high degree of comorbidity [29, 30]. The inflammatory hypothesis suggests that inflammatory responses caused by abnormal cytokines [31, 32] and excessive immune activation [33, 34] are involved in mental disorders' occurrence and development. Studies have confirmed that anxiety-related psychological stress can activate inflammatory responses and is associated with increased circulating inflammatory markers [35–37]. Studies have shown a significant increase in the concentration of IL-6 and CRP in the peripheral blood of anxiety disorder patients [38–41]. However, some studies have reached different conclusions. Wagner et al. found that the CRP serum level in anxiety disorders was not different from a simple anxiety disorder group and that the IL-6 level in anxiety disorder patients was lower than that in the simple anxiety disorder group [42].

In this study, we focused on whether peripheral blood IL-6 and hs-CRP can predict the occurrence of CHD in patients with anxiety disorders. The results indicated that both IL-6 and hs-CRP were risk factors for CHD-combined anxiety disorders. IL-6 and hs-CRP were still independent risk factors for CHD-combined anxiety disorders even after adjusting for common risk factors such as sex, age, smoking status, diabetes mellitus, and hypertension. This study found that patients with inflammation complicated by anxiety disorder complicated by CHD responded significantly more than patients with simple anxiety disorder, which may cause high mortality and poor prognosis in patients with coronary heart disease complicated by an anxiety disorder. The results from the Spearman correlation analysis in this study also showed that elevated hs-CRP was positively correlated with the degree of coronary artery stenosis combined with anxiety disorders, further supporting the possibility of hs-CRP as a risk factor for CHD with anxiety disorders.

Hcy is an amino acid with biological functions in vivo methionine metabolism. It mediates methylation and plays a key role in central nervous system biochemical balance [43]. Current studies showed elevated Hcy is associated with low-grade inflammation [44] and can increase the risk of coronary artery disease in adults [45]. Recent studies have shown that elevated Hcy can promote lipid deposition in foam cells and accelerate the progression of atherosclerosis [46]. Clinical studies have found that the plasma expression of Hcy is elevated in CHD [47, 48] and is related to coronary artery stenosis degree [49]. Therefore, Hcy can predict major adverse cardiovascular events and has important clinical significance in determining the condition and prognosis of CHD patients [47]. However, there are few studies on the changes in peripheral blood levels of Hcy in patients with anxiety disorders, and the results are inconsistent. Studies have shown no difference in serum Hcy levels between people with anxiety disorders and healthy individuals. [49]. Another study found that adolescents' severity of anxiety disorders was positively correlated with serum Hcy concentration [11]. We found that Hcy was also an independent risk factor for CHD in patients with anxiety disorders after adjusting for related risk factors. Spearman correlation analysis also confirmed that Hcy level was positively correlated to coronary artery stenosis degree-combined anxiety disorders, suggesting its potential value as a biomarker for predicting CHD.

In this study, hs-CRP had high specificity (88%) but low sensitivity (47%) in predicting CHD in patients with anxiety disorders. These findings are inconsistent with the high sensitivity of hs-CRP in predicting CHD reported by Tajfard et al. [17]. Similarly, Hcy also had high specificity (85%) but low sensitivity (48%) in predicting CHD in patients with anxiety disorders. Considering the intrinsic correlation of anxiety disorder with hs-CRP and Hcy, we believe this phenomenon may be related to all participants in our study having anxiety disorders. In addition, we did not adjust for those traditional risk factors when calculating sensitivity to increase clinical practicability. This also led to a decrease in sensitivity to some extent. The results of the ROC curve analysis suggested that hs-CRP combined with Hcy had a significantly larger AUC for the prediction of CHD in patients with anxiety disorders than did hs-CRP or Hcy alone. Using the inflammatory cytokine hs-CRP and the metabolic factor Hcy together to predict CHD in patients with anxiety disorders is more comprehensive and accurate than using hs-CRP or Hcy alone. When hs-CRP was ≤2.0 mg/L, and Hcy was ≤11.96 *μ*mol/L, patients with anxiety disorders were highly unlikely to have CHD, with a high negative predictive value for determining whether patients with anxiety disorders admitted to the hospital due to chest pain are complicated with CHD and with important clinical significance. Because these indicators are easy and inexpensive to measure, the potential surgical risks and waste of medical resources can be avoided to a certain extent for patients with anxiety disorders who strongly require CAG. In addition, significantly elevated IL-6, hs-CRP, or Hcy levels in the peripheral blood of patients with anxiety disorders also suggest a CHD risk.

This study also has some shortcomings. First, the sample size is small, the representativeness of the samples is low, and the results are inevitably biased. It is necessary to conduct larger studies to validate our results and to define the best predictors more rigorously. Second, the HAMA is used to determine patient's anxiety status, which is simple and commonly used in clinical practice. However, like other evaluation methods for determining anxiety disorders, the HAMA inevitably has evaluation bias. Therefore, the possibility of these biases affecting the study results cannot be ruled out. Third, anxiety disorder complicated by CHD is affected by many factors, and it is unlikely that all of these possible variables were included in the study. Fourth, we could not obtain the specific values of IL-6 for all subjects due to the sensitivity of the detection reagents; therefore, we only divided them into high and low IL-6 groups based on the IL-6 test results. This approach made it impossible to obtain the optimal cutoff value and predictive value of IL-6 for predicting CHD in anxiety disorder patients.

## 5. Conclusion

We determined that IL-6, hs-CRP, and Hcy were independent risk factors for CHD with anxiety disorders. hs-CRP and Hcy serum levels have high clinical predictive value, especially negative predictive value, in assessing whether patients with anxiety disorders are complicated with CHD. The combined detection of hs-CRP and Hcy can play a better predictive role, providing a clinical basis for the noninvasive prediction of CHD in patients with anxiety disorders.

## Figures and Tables

**Figure 1:** ROC curves for hs-CRP, Hcy, and their combined detection for predicting CHD in patients with anxiety disorders. ^∗^*P* < 0.05 vs. hs-CRP/Hcy for AUC.

**Table 1:** Characteristics between patients with anxiety disorders complicated with CHD or not.

Parameters	Patients with anxiety disorders complicated with CHD (*n* = 64)	Patients with anxiety disorders alone (*n* = 89)	*P* value
HAMA score	16.5 (15, 18.75)	16 (15, 19.5)	0.702^a^
Male	41 (64.1%)	36 (40.4%)	0.004^b^
Age (years)	64 (58.0, 69.75)	62.0 (56.0, 65.0)	0.024^a^
Smoking	23 (35.9%)	14 (15.7%)	0.004^b^
Diabetes mellitus	23 (35.9%)	15 (16.9%)	0.007^b^
Hypertension	42 (65.6%)	39 (43.8%)	0.008^b^
BMI (kg/m^2^)	25.31 (23.66, 27.75)	24.21 (22.85, 26.53)	0.063^a^
IL-6 (≥3.5 pg/mL)	25 (39.1%)	8 (9.0%)	<0.001^b^
hs-CRP (mg/L)	1.76 (0.70, 4.28)	0.84 (0.45, 1.66)	<0.001^a^
Hcy (*μ*mol/L)	11.49 (9.66, 16.28)	10.08 (8.42, 11.43)	<0.001^a^
Fibrinogen (g/L)	2.73 ± 0.45	2.67 ± 0.47	0.459^c^
D-dimer (g/L)	0.24 (0.19, 0.29)	0.22 (0.18, 0.26)	0.112^a^
Cortisol (nmol/L)	309.38 ± 90.28	307.36 ± 93.33	0.894^c^
Norepinephrine (nmol/L)	0.41 (0.26, 0.53)	0.37 (0.29, 0.52)	0.814^a^
tCholesterol (mmol/L)	5.10 (4.52, 5.74)	4.97 (4.20, 5.60)	0.155^a^
HDL-C (mmol/L)	1.11 ± 0.32	1.17 ± 0.25	0.222^c^
LDL-C (mmol/L)	3.00 ± 0.79	2.86 ± 0.87	0.314^c^
Triglyceride (mmol/L)	1.56 (1.12, 2.20)	1.39 (0.98, 2.17)	0.141^a^
Lp(a) (mmol/L)	152.58 (58.92, 294.15)	107.35 (51.09, 208.87)	0.207^a^
ApoB (mmol/L)	1.12 ± 0.28	1.05 ± 0.27	0.104^c^
Creatinine (*μ*mol/L)	64.15 (55.8, 71.78)	60.1 (55.1, 68.7)	0.116^a^

Notes: data are shown as mean ± SD, median with IQR, or absolute number (percentage). ^a^Student *t*-test; ^b^chi-square test; ^c^Mann-Whitney *U* test. Abbreviations: CHD: coronary heart disease; HAMA: Hamilton Anxiety Scale; BMI: body mass index; IL-6: interleukin-6; hs-CRP: high-sensitivity C-reactive protein; Hcy: homocysteine; tCholesterol: total cholesterol; HDL-C: high-density lipoprotein cholesterol; LDL-C: low-density lipoprotein cholesterol; Lp(a): lipoprotein (a); ApoB: apolipoprotein B.

**Table 2:** Risk factors for CHD in patients with anxiety disorder.

Risk factors	Univariable analysis		Multivariable analysis	
	OR (95% CI)	*P* value	OR (95% CI)	*P* value
Male	0.381 (0.196~0.740)	0.004	0.491 (0.197~1.225)	0.127
Age	1.046 (1.004~1.090)	0.031	1.038 (0.987~1.092)	0.143
Smoking	0.333 (0.155~0.716)	0.005	0.446 (0.162~1.228)	0.118
Diabetes mellitus	0.361 (0.170~0.768)	0.008	0.395 (0.160~0.971)	0.043
Hypertension	0.381 (0.195~0.744)	0.005	0.584 (0.195~0.744)	0.183
IL-6 (≥3.5 pg/mL)	0.154 (0.064~0.373)	<0.001	0.194 (0.064~0.373)	0.001
hs-CRP	1.386 (1.156~1.662)	<0.001	1.266 (1.156~1.662)	0.017
Hcy	1.220 (1.101~1.351)	<0.001	1.185 (1.101~1.351)	0.006

Note: results of binary logistic regression analysis are presented as adjusted OR, 95% CI, and *P* value. Abbreviations: CHD: coronary heart disease; IL-6: interleukin -6; hs-CRP: high-sensitivity C-reactive protein; Hcy: homocysteine; OR: odds ratio; CI: confidence interval.

## Data Availability

The datasets used and analyzed during the current study are available from the corresponding author upon reasonable request.

## Abbreviations

CHD: Coronary heart disease
CAG: Coronary angiography
BMI: Body mass index
IL-6: Interleukin -6
Hs-CRP: High-sensitivity C-reactive protein
Hcy: Homocysteine
ROC: Receiver operating characteristic
HAMA: Hamilton Anxiety Scale
HDL-C: High-density lipoprotein cholesterol
LDL-C: Low-density lipoprotein cholesterol
IQR: Interquartile range
AUC: Area under the curve
OR: Odds ratio
CI: Confidence interval.

## References

[1] Behrens T., Heidrich J., Keil U. (2015). Modifying behaviors in patients with coronary heart disease. *Deutsches Ärzteblatt International*.

[2] Han S. S., Wang Q., Li D., Wang S. Q. (2019). Effect of pravastatin combined with metoprolol on cardiac function, glycolipid metabolism and other related indicators in patients with diabetes mellitus complicated with coronary heart disease. *Journal of Molecular Diagnostics and Therapy*.

[3] He Y. Z., Huang C. Y., Huang J. W., Li L. J., Liang S., Wang Q. G. (2019). Based on the intestinal micro-ecosystem, the spleen theory is discussed in the treatment of coronary heart disease. *Journal of Liaoning University of Traditional Chinese Medicine*.

[4] Huang G. C., Hu X., Tang Y. Q., Tan J. Y., Zhou F., Feng N. N. (2019). Research advances related to homocysteine and Alzheimer's disease. *Public Health and Preventive Medicine*.

[5] Purves K. L., Coleman J. R. I. (2020). A major role for common genetic variation in anxiety disorders. *Molecular Psychiatry*.

[6] Roest A. M., Martens E. J., de Jonge P., Denollet J. (2010). Anxiety and risk of incident coronary heart disease: a meta-analysis. *Journal of the American College of Cardiology*.

[7] Whooley M. A., de Jonge P., Vittinghoff E. (2008). Depressive symptoms, health behaviors, and risk of cardiovascular events in patients with coronary heart disease. *JAMA*.

[8] Celano C. M., Daunis D. J., Lokko H. N., Campbell K. A., Huffman J. C. (2016). Anxiety disorders and cardiovascular disease. *Current Psychiatry Reports*.

[9] Crum-Cianflone N. F., Bagnell M. E., Schaller E. (2014). Impact of combat deployment and posttraumatic stress disorder on newly reported coronary heart disease among US active duty and reserve forces. *Circulation*.

[10] Herbison P., Tie C. L., Tang E., Bermingham B., Wong C. K. (2015). Components of depression and 6-year mortality after an acute coronary syndrome. *The American Journal of Medicine*.

[11] Cohen B. E., Edmondson D., Kronish I. M. (2015). State of the art review: depression, stress, anxiety, and cardiovascular disease. *American Journal of Hypertension*.

[12] Tully P. J., Harrison N. J., Cheung P., Cosh S. (2016). Anxiety and cardiovascular disease risk: a review. *Current Cardiology Reports*.

[13] Zhang T., Xie X., Li Q. (2022). Hypogyrification in generalized anxiety disorder and associated with insomnia symptoms. *Sleep*.

[14] Cagney D. N., Sul J., Huang R. Y., Ligon K. L., Wen P. Y., Alexander B. M. (2018). The FDA NIH biomarkers, EndpointS, and other Tools (BEST) resource in neuro-oncology. *Neuro-Oncology*.

[15] Marcos-Jubilar M., Orbe J. (2021). Association of SDF1 and MMP12 with atherosclerosis and inflammation. *Clinical and Experimental Study*.

[16] Ridker P. M., Everett B. M., Thuren T. (2017). Antiinflammatory therapy with canakinumab for atherosclerotic disease. *The New England Journal of Medicine*.

[17] Tajfard M., Tavakoly Sany S. B., Avan A. (2019). Relationship between serum high sensitivity C-reactive protein with angiographic severity of coronary artery disease and traditional cardiovascular risk factors. *Journal of Cellular Physiology*.

[18] Tajfard M., Latiff L. A., Rahimi H. R. (2017). Serum concentrations of MCP-1 and IL-6 in combination predict the presence of coronary artery disease and mortality in subjects undergoing coronary angiography. *Molecular and Cellular Biochemistry*.

[19] Mauer J., Denson J. L., Brüning J. C. (2015). Versatile functions for IL-6 in metabolism and cancer. *Trends in Immunology*.

[20] Libby P. (2021). Targeting inflammatory pathways in cardiovascular disease: the inflammasome, interleukin-1, interleukin-6 and beyond. *Cell*.

[21] Held C., White H. D., Stewart R. A. H. (2017). Inflammatory biomarkers interleukin-6 and C-reactive protein and outcomes in stable coronary heart disease: experiences from the STABILITY (Stabilization of Atherosclerotic Plaque by Initiation of Darapladib Therapy) trial. *Journal of the American Heart Association*.

[22] Castro A. R., Silva S. O., Soares S. C. (2018). The use of high sensitivity C-reactive protein in cardiovascular disease detection. *Journal of pharmacy & pharmaceutical sciences: a publication of the Canadian Society for Pharmaceutical Sciences, Societe canadienne des sciences pharmaceutiques*.

[23] Sara J. D. S., Prasad M., Zhang M. (2017). High-sensitivity C-reactive protein is an independent marker of abnormal coronary vasoreactivity in patients with non-obstructive coronary artery disease. *American Heart Journal*.

[24] Tayefi M., Tajfard M., Saffar S. (2017). hs-CRP is strongly associated with coronary heart disease (CHD): a data mining approach using decision tree algorithm. *Computer Methods and Programs in Biomedicine*.

[25] Kinoshita A., Onoda H., Imai N., Nishino H., Tajiri H. (2015). C-reactive protein as a prognostic marker in patients with hepatocellular carcinoma. *Hepato-Gastroenterology*.

[26] Li H., Sun K., Zhao R. (2018). Inflammatory biomarkers of coronary heart disease. *Frontiers in Bioscience (Scholar Edition)*.

[27] Volanakis J. E. (2001). Human C-reactive protein: expression, structure, and function. *Molecular Immunology*.

[28] Stapp J. M., Sjoelund V., Lassiter H. A., Feldhoff R. C., Feldhoff P. W. (2005). Recombinant rat IL-1*β* and IL-6 synergistically enhance C3 mRNA levels and complement component C3 secretion by H-35 rat hepatoma cells. *Cytokine*.

[29] Penninx B. W., Pine D. S., Holmes E. A., Reif A. (2021). Anxiety disorders. *Lancet*.

[30] Kaufman J., Charney D. (2000). Comorbidity of mood and anxiety disorders. *Depression and Anxiety*.

[31] Schiepers O. J., Wichers M. C., Maes M. (2005). Cytokines and major depression. *Progress in Neuro-Psychopharmacology & Biological Psychiatry*.

[32] Michopoulos V., Powers A., Gillespie C. F., Ressler K. J., Jovanovic T. (2017). Inflammation in fear- and anxiety-based disorders: PTSD, GAD, and beyond. *Neuropsychopharmacology: official publication of the American College of Neuropsychopharmacology*.

[33] Luo Y., He H., Zhang M., Huang X., Fan N. (2016). Altered serum levels of TNF-*α*, IL-6 and IL-18 in manic, depressive, mixed state of bipolar disorder patients. *Psychiatry Research*.

[34] Luo Y., He H., Zhang J., Ou Y., Fan N. (2019). Changes in serum TNF-*α*, IL-18, and IL-6 concentrations in patients with chronic schizophrenia at admission and at discharge. *Comprehensive Psychiatry*.

[35] Furtado M., Katzman M. A. (2015). Neuroinflammatory pathways in anxiety, posttraumatic stress, and obsessive compulsive disorders. *Psychiatry Research*.

[36] Steptoe A., Hamer M., Chida Y. (2007). The effects of acute psychological stress on circulating inflammatory factors in humans: a review and meta-analysis. *Brain, Behavior, and Immunity*.

[37] Tayefi M., Shafiee M., Kazemi-Bajestani S. M. R. (2017). Depression and anxiety both associate with serum level of hs-CRP: a gender-stratified analysis in a population-based study. *Psychoneuroendocrinology*.

[38] Zou Z., Zhou B., Huang Y., Wang J., Min W., Li T. (2020). Differences in cytokines between patients with generalised anxiety disorder and panic disorder. *Journal of Psychosomatic Research*.

[39] Tang Z., Ye G., Chen X. (2018). Peripheral proinflammatory cytokines in Chinese patients with generalised anxiety disorder. *Journal of Affective Disorders*.

[40] Naudé P. J. W., Roest A. M., Stein D. J., de Jonge P., Doornbos B. (2018). Anxiety disorders and CRP in a population cohort study with 54,326 participants: the LifeLines study. *The world journal of biological psychiatry: the official journal of the World Federation of Societies of Biological Psychiatry*.

[41] Costello H., Gould R. L., Abrol E., Howard R. (2019). Systematic review and meta-analysis of the association between peripheral inflammatory cytokines and generalised anxiety disorder. *BMJ Open*.

[42] Wagner E. N., Strippoli M. F., Ajdacic-Gross V. (2020). Generalized anxiety disorder is prospectively associated with decreased levels of Interleukin-6 and adiponectin among individuals from the community. *Journal of Affective Disorders*.

[43] Folstein M., Liu T., Peter I. (2007). The homocysteine hypothesis of depression. *The American Journal of Psychiatry*.

[44] Jonasson T., Ohlin A. K., Gottsäter A., Hultberg B., Ohlin H. (2005). Plasma homocysteine and markers for oxidative stress and inflammation in patients with coronary artery disease--a prospective randomized study of vitamin supplementation. *Clinical Chemistry and Laboratory Medicine*.

[45] Ganguly P., Alam S. F. (2015). Role of homocysteine in the development of cardiovascular disease. *Nutrition Journal*.

[46] Guo W., Zhang H., Yang A. (2020). Homocysteine accelerates atherosclerosis by inhibiting scavenger receptor class B member1 via DNMT3b/SP1 pathway. *Journal of Molecular and Cellular Cardiology*.

[47] Cheng M., Cheng M., Wei Q. (2020). Association of myeloperoxidase, homocysteine and high-sensitivity C-reactive protein with the severity of coronary artery disease and their diagnostic and prognostic value. *Experimental and Therapeutic Medicine*.

[48] Guan J., Wu L., Xiao Q., Pan L. (2021). Levels and clinical significance of serum homocysteine (Hcy), high-density lipoprotein cholesterol (HDL-C), vaspin, and visfatin in elderly patients with different types of coronary heart disease. *Annals of palliative medicine*.

[49] Bjelland I., Tell G. S., Vollset S. E., Refsum H., Ueland P. M. (2003). Folate, vitamin B12, homocysteine, and the MTHFR 677C→T polymorphism in anxiety and depression. *Archives of General Psychiatry*.

